The article "Dynamic contrast‐enhanced MRI perfusion for differentiating between melanoma and lung cancer brain metastases" was published in 2017. Journal: Cancer Med.

# Dynamic contrast‐enhanced MRI perfusion for differentiating between melanoma and lung cancer brain metastases

**DOI:** 10.1002/cam4.1046

**Published:** 2017-03-17

**Authors:** Vaios Hatzoglou, Jamie Tisnado, Alpesh Mehta, Kyung K. Peck, Mariza Daras, Antonio M. Omuro, Kathryn Beal, Andrei I. Holodny

**Affiliations:** ^1^ Department of RadiologyMemorial Sloan Kettering Cancer CenterNew York CityNew York; ^2^ Brain Tumor CenterMemorial Sloan Kettering Cancer CenterNew York CityNew York; ^3^ Department of Medical PhysicsMemorial Sloan Kettering Cancer CenterNew York CityNew York; ^4^ Department of NeurologyMemorial Sloan Kettering Cancer CenterNew York CityNew York; ^5^ Department of Radiation OncologyMemorial Sloan Kettering Cancer CenterNew York CityNew York

**Keywords:** Brain tumors, melanoma, neuroimaging, non‐small cell lung cancer, perfusion weighted MRI

## Abstract

Brain metastases originating from different primary sites overlap in appearance and are difficult to differentiate with conventional MRI. Dynamic contrast‐enhanced (DCE)‐MRI can assess tumor microvasculature and has demonstrated utility in characterizing primary brain tumors. Our aim was to evaluate the performance of plasma volume (*V*p) and volume transfer coefficient (*K* ^trans^) derived from DCE‐MRI in distinguishing between melanoma and nonsmall cell lung cancer (NSCLC) brain metastases. Forty‐seven NSCLC and 23 melanoma brain metastases were retrospectively assessed with DCE‐MRI. Regions of interest were manually drawn around the metastases to calculate *V*p_mean_ and $K_{\mathrm{mean}}^{\mathrm{trans}}$. The Mann–Whitney *U* test and receiver operating characteristic analysis (ROC) were performed to compare perfusion parameters between the two groups. The *V*p_mean_ of melanoma brain metastases (4.35, standard deviation [SD] = 1.31) was significantly higher (*P* = 0.03) than *V*p_mean_ of NSCLC brain metastases (2.27, SD = 0.96). The $K_{\mathrm{mean}}^{\mathrm{trans}}$ values were higher in melanoma brain metastases, but the difference between the two groups was not significant (*P* = 0.12). Based on ROC analysis, a cut‐off value of 3.02 for *V*p_mean_ (area under curve = 0.659 with SD = 0.074) distinguished between melanoma brain metastases and NSCLC brain metastases (*P* < 0.01) with 72% specificity. Our data show the DCE‐MRI parameter *V*p_mean_ can differentiate between melanoma and NSCLC brain metastases. The ability to noninvasively predict tumor histology of brain metastases in patients with multiple malignancies can have important clinical implications.

## Introduction

Brain metastases occur more frequently than primary brain tumors and represent one of the most common neurologic complications of cancer 1, 2. The incidence of brain metastases ranges from 9% to 17% based on various studies 2 and there are >170,000 new cases per year in the United States 3. A rise in the number of cases is expected as a result of several factors, including better imaging quality and accessibility and the increased prevalence of individuals living with cancer due to improved systemic control 2, 3. In addition, many cancer survivors develop a second malignancy that is new and unrelated to their original cancer 4. The number of patients with second and high‐order malignancies is growing 5 and second cancers have been reported to comprise up to 18% of all incident cancers in the United States, superseding first primary cancers of the lung, breast, and prostate 6. As a result of these trends, the development of new brain metastases in a patient with a history of two or more different cancers is becoming a more common clinical scenario 7, 8.

Accurately predicting the histology of brain metastases in a patient with multiple cancers without resorting to craniotomy has important clinical implications such as correct staging of the primary tumor and selecting the most effective treatment regimen, both of which impact patient survival. Conventional anatomy‐based MRI provides valuable information regarding the size, number, and location of brain metastases, but is limited in terms of differentiating between histologic subtypes because brain metastases demonstrate similar characteristics on conventional MR imaging 9.

Dynamic contrast‐enhanced (DCE)‐MRI is an advanced imaging technique that has recently demonstrated promise for distinguishing between different primary brain tumor histologies 10. Unlike conventional imaging, DCE‐MRI can quantitatively assess tumor microvasculature by measurement of a range of parameters that reflect specific physiologic characteristics such as plasma volume (*V*p) and volume transfer coefficient (*K* ^trans^).

Lung cancer, breast cancer, and melanoma account for 67–80% of all cancers and are the most frequent to develop brain metastases 2, 11. The aim of our study was to evaluate the ability of DCE‐MRI to differentiate between non‐small cell lung cancer (NSCLC) and melanoma brain metastases. Lung cancer metastases are considered hypovascular while melanoma is typically hypervascular 12, 13. We hypothesized that *V*p would be an accurate predictor of histology and more elevated in melanoma than NSCLC brain metastases since *V*p provides an estimate of tumor microvascular density 14, 15.

## Methods

This retrospective study was performed at a tertiary cancer institution in accordance with the Health Insurance Portability and Accountability Act and with local Institutional Review Board approval, including waiver of informed consent.

### Eligibility

We queried institutional and departmental databases for consecutive patients with either NSCLC or melanoma brain metastases scheduled for treatment with stereotactic radiosurgery (SRS) or partial brain radiation therapy (pBRT) from January 2012 through March 2013 and who had pre‐radiotherapy DCE‐MRI. All eligible patients had biopsy proven melanoma or NSCLC based on tissue samples acquired from the primary tumors and/or extracranial metastases. Biopsies of the intracranial lesions were not deemed necessary based on the clinical presentations of these patients with Stage IV disease and imaging findings that were typical for brain metastases. We excluded brain metastases that were previously resected and/or irradiated. Any metastases that were almost entirely cystic or necrotic were also excluded. Patients who were actively being treated with anti‐angiogenic agents or steroids were excluded as well because of the potential confounding impact of these drugs on the innate perfusion characteristics of the metastases. Finally, patients with a second primary malignancy in addition to NSCLC or melanoma were excluded to minimize the possibility of the brain lesions having originated from another source.

### DCE‐MRI acquisition and analysis

Patients were scanned on 1.5T or 3T scanners (Signa Excite, HDx and Discovery 750, GE Healthcare, Milwaukee, WI) using an 8‐channel head coil. Standard T1‐weighted, T2‐weighted, diffusion‐weighted, fluid‐attenuated inversion recovery, susceptibility‐weighted, and contrast T1‐weighted images were acquired in multiple planes. The precontrast T1‐weighted and T2‐weighted images of the melanoma and NSCLC brain metastases were assessed in a blinded fashion by a board‐certified attending neuroradiologist with 10 years of neuroimaging experience. The metastases were scored as hypointense, isointense, or hyperintense on each sequence.

Gadopentetate dimeglumine (Magnevist; Bayer HealthCare Pharmaceuticals, Wayne, NJ) was power‐injected via an intravenous catheter (18–21 gauge) at doses standardized by patient body weight (0.2 mL/kg body weight, maximum 20 mL) at 2–3 mL/s. T1‐weighted DCE perfusion data were acquired using an axial 3D SPGR (Spoiled Gradient Recalled Echo) sequence (TR, 4–5 ms; TE, 1–2 ms; section thickness, 5 mm; flip angle, 25°; FOV, 24 cm; matrix, 256 × 128). Ten phases were acquired pre‐injection followed by another 30 phases during the dynamic injection of intravenous contrast. This was followed by a 40‐mL saline flush. The time between phases (temporal resolution) was 5–6 sec. Matching post contrast T1‐weighted (TR/TE, 600/8 ms; thickness, 5 mm; matrix, 256 × 224) spin‐echo images were obtained. Ten to twelve slices were obtained for the DCE color maps and matching T1 post contrast images. The native T1 was not measured and a fixed baseline value of 1000 ms was utilized.

An off‐line workstation with available commercial imaging analysis software (NordicICE; Nordic Neuro Lab, Bergen, Norway) was used to process all raw perfusion data. Perfusion data preprocessing consisted of noise reduction, motion artifact rectification, and semi‐automatic selection of arterial input function (AIF) from the middle cerebral artery. Curves displaying an optimal relationship between AIF and concentration‐time curve were carefully chosen. We used a two‐compartment model with kinetic modeling and AIF‐based vascular deconvolution as proposed by Murase 16 to calculate the pharmacokinetic parameters plasma volume (*V*p) and volume transfer coefficient (*K* ^trans^). A region of interest (ROI) encompassing the entire tumor was manually drawn on the single transaxial slice representing the largest sum of the bi‐dimensional size measurements for each metastasis. Large vessels were excluded from the ROI in order not to bias measurements. The ROIs were then transferred onto the matching *V*p and *K* ^trans^ perfusion maps and the *V*p_mean_ and $K_{\mathrm{mean}}^{\mathrm{trans}}$ values for each lesion were measured and recorded. A board‐certified attending neuroradiologist with 10 years of neuroimaging experience approved all ROIs and was blinded to lesion histology.

### Statistical analysis

A Mann–Whitney *U* test was used to assess the differences between the DCE‐MRI pharmacokinetic parameters (*V*p_mean_ and $K_{\mathrm{mean}}^{\mathrm{trans}}$). A *P* < 0.05 was considered statistically significant. Receiver operating characteristic (ROC) curve analysis was performed using Statistical Package for the Social Sciences Statistics (Version 22; IBM, Armonk, NY) to determine which cut‐off values provided the best combination of sensitivity and specificity for differentiating between melanoma and NSCLC brain metastases. Fisher's exact test was used assess the differences in T1‐weighted and T2‐weighted signal characteristics between the melanoma and NSCLC metastases. A *P* < 0.05 was considered statistically significant.

## Results

### Patient characteristics

A total of 56 consecutive patients (31 male and 25 female) with a mean age of 66.4 (range, 43–91) years were included in the study. Of these, there were 37 NSCLC patients with 47 brain metastases and 19 melanoma patients with 23 brain metastases for a total of 70 lesions evaluated with DCE‐MRI prior to SRS or pBRT. The maximum dimensions of the lesions ranged from 0.5 cm to 5.1 cm on axial T1‐weighted post contrast imaging.

### Pharmacokinetic parameters

The *V*p_mean_ for melanoma brain metastases was significantly higher (*P* = 0.03) than *V*p_mean_ for NSCLC brain metastases. Specifically, the *V*p_mean_ for melanoma brain metastases was 4.35 (standard deviation [SD] = 1.31; range: 0.38–17.16) and *V*p_mean_ for NSCLC brain metastases was 2.27 (SD = 0.96; range: 0.08–5.19). This is summarized in Figure 1. Representative images from two patients are provided in Figure 2. The $K_{\mathrm{mean}}^{\mathrm{trans}}$ values were higher in melanoma (mean = 0.07, SD = 0.02) compared to NSCLC (mean = 0.04, SD = 0.01), but the difference between the groups was not significant (*P* = 0.12).

**Figure 1:** Box plot illustrating the mean values and standard deviations for *V*p_mean_ of non‐small cell lung cancer (NSCLC) and melanoma brain metastases.

**Figure 2:** Axial T1‐weighted postcontrast images (A and C) with corresponding *V*p perfusion color maps (B and D) of right frontal lobe (arrows) melanoma (top row) and right frontal lobe (arrows) NSCLC (bottom row) brain metastases. The melanoma brain metastasis demonstrates greater elevation of *V*p (*V*p_mean_ = 8.46) than the lung cancer brain metastasis (*V*p_mean_ = 1.52).

### ROC analysis

Based on ROC analysis, a cut‐off value of 3.02 for *V*p_mean_ (area under curve = 0.659 with SD = 0.074) distinguished between melanoma brain metastases and NSCLC brain metastases (*P* < 0.01) with 72% specificity (Fig. 3).

**Figure 3:** Receiver operating characteristic (ROC) curve depicting the true‐positive rate (specificity) and the false‐positive rate (sensitivity) of the pharmacokinetic parameter *V*p in differentiating NSCLC and melanoma brain metastases.

### Conventional T1‐weighted and T2‐weighted signal

Eight of 23 (35%) melanoma brain metastases demonstrated T1 hyperintense signal. Thirteen of 47 (28%) NSCLC brain metastases demonstrated T1 hyperintense signal. The difference between the two groups was not statistically significant (*P* = 0.58). The remaining melanoma and NSCLC lesions were hypointense on T1 with the exception of two isointense NSCLC metastases. Five of 23 (22%) melanoma brain metastases demonstrated T2 hypointense signal compared to nine of 47 (19%) NSCLC brain metastases. The difference between the groups was not statistically significant (*P* = 0.99). The remaining lesions were all T2 hyperintense.

## Discussion

In this study, we found the pharmacokinetic variable *V*p_mean_ derived from DCE‐MRI was significantly more elevated in brain metastases originating from melanoma (*V*p_mean_ = 4.35) than brain metastases from NSCLC (*V*p_mean_ = 2.27). The ability to noninvasively distinguish between brain metastases from different primary sites is becoming more important as the incidence of brain metastases and numbers of patients developing secondary malignancies both continue to rise 2, 3, 5. Patients with a personal history of two or more malignancies and new brain metastases are increasingly common at our high volume cancer center and in the community at large 7, 8. It is often unclear from which primary site the brain metastases have originated based on conventional MRI and these patients are therefore frequently subjected to invasive neurosurgery, with all its inherent costs and risks, for accurate tumor staging. Correctly identifying the histopathology of intracranial metastatic disease has major treatment implications. Patients with brain metastases are being treated on a more individualized basis 17 because knowledge of tumor biology has improved and greater selections of biologically targeted systemic agents are currently available 1.

Conventional MRI is a very useful tool for the detection of brain metastases but cannot readily differentiate between tumor histologies. Brain metastases are typically nodular, iso‐ or hypointense on T1‐weighted imaging, hyperintense on T2‐weighted imaging, and avidly enhance after contrast administration regardless of their primary site of origin 9. Even the presence of hemorrhage which is classically associated with brain metastases from melanoma, choriocarcinoma, renal cell cancer, and thyroid cancer, is not a reliable clue regarding site of origin because hemorrhagic brain metastases are most frequently from lung and breast cancer due to their overall higher prevalence 9.

MRI perfusion is an advanced imaging technique that allows for quantitative assessment of tumor microvasculature by analyzing the distribution kinetics of an intravenously injected low‐molecular‐weight paramagnetic agent in the microvessels and extravascular‐extracellular space of tissue under review. *V*p derived from DCE‐MRI is defined as the blood plasma volume per unit volume of tissue and is the physiologic equivalent of relative cerebral blood volume (rCBV) obtained from dynamic susceptibility‐weighted contrast‐enhanced (DSC) perfusion imaging. *V*p and rCBV correlate with histologic and angiographic assessment of vascular density in human brain tumors 15, 18, 19 and have been successfully utilized by us and other research groups to predict grading in gliomas 20, 21, 22 and to differentiate between hypervascular and hypovascular metastases to the spine 23.

There are currently no established imaging biomarkers for distinguishing between brain metastases from different primary tumors. Several groups of investigators that assessed the potential of perfusion imaging for this purpose have generated mixed results 24, 25, 26, 27. These prior endeavors included smaller and more heterogeneous sample sizes of brain metastases ranging from 20 to 36 in total compared to 70 lesions (47 melanoma and 23 NSCLC) for our study. Kremer et al. 24 reported that mean rCBV_max_ measurements of melanoma and renal carcinoma brain metastases were significantly greater than mean rCBV_max_ of lung cancer brain metastases. The ratio of melanoma rCBV_max_ to lung cancer rCBV_max_ was 1.8 (5.35/2.94), which is comparable to the ratio of 1.9 (4.35/2.27; melanoma/NSCLC) we discovered for *V*p_mean_. The authors of that study did not specify if the lung cancer brain metastases assessed were from NSCLC, small cell carcinoma, or a combination of both.

Hakyemez et al. 25 did not find a statistically significant difference between the rCBV values of 16 lung and seven breast cancer metastases. This result is possibly related to lung and breast cancer metastases both being typically hypovascular and therefore overlapping in their perfusion imaging characteristics 12, 23 or secondary to inherent limitations of the DSC technique. The rCBV measurements derived from DSC are semiquantitative and can be influenced by multiple postprocessing steps, including the choice of normal contralateral white matter and correction technique to address contrast extravasation 28, 29. Additional drawbacks of DSC perfusion imaging include sensitivity to susceptibility effects from bone, calcification, and hemorrhage 30. DCE‐MRI perfusion is less sensitive to susceptibility artifacts and *V*p has been demonstrated to be superior to rCBV for quantitative evaluation of cerebral blood volume 31.

A study by Dolgushin et al. 26 prospectively examined different CT perfusion parameters of 36 brain metastases and revealed that lesions from different primaries can be differentiated from each other in 57% of cases. The utilization of CT for evaluation of brain metastases can be helpful if MRI is unavailable or contraindicated, but MRI is recognized as the reference standard and has been shown to be more sensitive than CT by multiple studies 32, 33, 34. A recent investigation by Jung et al. 27 is similar to ours in that DCE‐MRI was used to evaluate the perfusion characteristics of hypervascular and hypovascular brain tumors, including glioblastomas and different types of metastases. Their subgroup comparison of 16 melanoma brain metastases to 16 typically hypovascular metastases (NSCLC, *n* = 7, breast = 6, colon = 3) did not demonstrate any significant difference between *K* ^trans^ and *V*p. Absence of difference in *K* ^trans^ matches our results and is expected since *K* ^trans^ measures the degree of contrast leakage from the intravascular to the extravascular compartment and brain metastases are inherently leakier than normal brain parenchyma regardless of primary site origin because they do not possess a blood‐brain barrier. The lack of difference in *V*p between the hypervascular and hypovascular brain lesions reported in their study is not in accord with our results and may be secondary to their smaller sample size (*n* = 32). The authors did find a statistically significant difference with quantitative analysis of the signal intensity time curves, which we did not assess.

Aside from its retrospective nature, our study had additional limitations. For example, the ROI for each metastasis was defined on a single axial image representing the largest sum of the lesion's bidimensional measurements rather than multiple slices to cover the entire tumor volume. This may have introduced a sampling error. We chose this technique because it is timely and clinically feasible even in a very busy oncology practice. Furthermore, many of the metastases in our study were smaller than 1.0 cm in the craniocaudal dimension and perfusion measurements from the adjacent slice may have been tainted by volume averaging with normal brain parenchyma or edema. The study results were also somewhat limited because there was some overlap in *V*p values between the two histologies and we could not differentiate NSCLC from melanoma with certainty in all cases. Lack of pathologic specimens directly from the metastases that were assessed with MRI perfusion is a limitation as well. Neurosurgical intervention was not practical in this patient population with stage IV disease. The differences in *V*p between melanoma and NSCLC brain metastases cannot, therefore, be definitively attributable to differences in vascular density. Another limitation is that we only included melanoma and NSCLC brain metastases. Our data cannot be generalized for patients with other types of brain metastases and cannot be utilized to predict the histology of brain metastases without knowledge of the primary tumors. Our goal in this study was to assess whether or not MRI perfusion could noninvasively predict the primary tumor site from which brain metastases originated in patients with two different known primary cancers (such as melanoma and NSCLC). We wanted to include at least 20 representative lesions from each histologic subtype that had undergone MRI perfusion in the pretreatment setting and this proved to be difficult with brain metastases from other primary sites. Melanoma and NSCLC brain metastases represent two of the most common types of brain metastases and those for which the greatest advances in targeted agents have been made in the past decade 1, 35, 36. We are currently accumulating more cases and intend to analyze breast cancer, renal cell cancer, and colorectal cancer brain metastases in addition to other less common histologies.

In conclusion, our study demonstrates that quantitative analysis of the DCE‐MRI parameter *V*p_mean_ can noninvasively differentiate between hypervascular (melanoma) and hypovascular (NSCLC) brain metastases in most cases. The application of this knowledge and continued exploration of advanced imaging for patients with brain metastases can have important and clinically relevant implications, particularly in our current era of increasing patient survival, cost containment, and personalized medicine. For example, *V*p from DCE‐MRI could potentially serve as an imaging biomarker to assess response in patients treated with anti‐angiogenic therapy and help determine treatment efficacy before structural changes become apparent on conventional MRI. Additional studies are needed to prospectively validate our results and to determine the impact of *V*p_mean_ in facilitating treatment planning for patients with a personal history of two malignancies and new brain metastases.

## Conflict of Interest

The authors have no conflicts of interest.
